# Tobacco Smoking Affects the Salivary Gram-Positive Bacterial Population

**DOI:** 10.3389/fpubh.2019.00196

**Published:** 2019-07-19

**Authors:** Ghiles Grine, Arthur Royer, Elodie Terrer, Ousmane Oumou Diallo, Michel Drancourt, Gérard Aboudharam

**Affiliations:** ^1^IHU Méditerranée Infection, Marseille, France; ^2^Aix-Marseille Université, IRD, MEPHI, IHU Méditerranée Infection, Marseille, France; ^3^Aix-Marseille Université, UFR Odontologie, Marseille, France

**Keywords:** tobacco smoking, *Streptococcus* spp, *Streptococcus australis*, oral fluid, gram-positive bacteria, culture

## Abstract

The microbial communities of the oral fluid are in direct contact with tobacco smoke, which may thus affect these communities. Few culture-based studies have analyzed the effects of tobacco smoking on the oral fluid microbiota. Using bacterial culture we investigated whether tobacco smoking altered the microbial diversity of the oral fluid, focusing on aerobic and facultative anaerobic Gram-positive bacteria otherwise comprising of major pathogens. Among 90 oral fluid specimens collected in 19 tobacco-smokers and 71 controls, the diversity did not significantly differ with age and with sex. However, diversity was significantly lower in tobacco-smokers (nine different species) than in non-smokers (18 different species) with all the species cultured in tabocco-smokers being also cultured in non-smokers. We isolated the human pathogen *Streptococcus australis* for the first time from oral fluid. Tobacco smoking significantly alters the saliva Gram-positive bacterial microbiota, including pathogens with potential implication in the pathogenesis of tobacco-related diseases such as periodontitis and peri-implantitis.

## Introduction

Saliva is a biological fluid secreted by the salivary glands into the oral cavity (1). The oral microbiome comprises an important bacterial diversity that is specific to each person and exhibits long-term stability over the years (2, 3). In particular, oral fluid is comprising of some Gram-positive bacteria implicated in infectious of the oral cavity along with infection distant from the oral cavity, such as infectious endocarditis (2). As the oral cavity is one of the gateways for pathogenic bacteria into the human body, there are different important interactions between the salivary microbiota, and other microbiota in the human body, especially the intestinal microbiota (1, 4). Also, several oral disorders and their treatment may have an impact on the bacterial diversity of the salivary microbiota (2). However, external factors may also affect microbial diversity in the salivary microbiota. Among these external factors, tobacco smoking has been shown to affect the oral microbiota (5, 6). Later studies however did not rely on culture (5), or were restricted to a few Gram-positive bacterial species (6).

Therefore, we specifically studied the potential impact of tobacco smoking on the Gram-positive oral bacterial flora at large to shed more light on the bacterial diversity of the salivary microbiome and its relation with external disorders, using culture.

## Materials and Methods

### Clinical Samples

This study has been approved by the Ethics Committee of the IHU Méditerranée Infection (N°2016–011). Accordingly, all the participants gave and signed an informed consent. A total of 90 saliva specimens were prospectively collected in individuals presenting at the Faculty of Odontology and the IHU Méditerranée Infection, located in Marseille, France. Salivary samples were collected using sterile swabs (Deltalab, Carcassonne, France) that were soaked in saliva after being rubbed into the oral cavity in the space between the buccal wall of the upper molar and also under the tongue. They were then deposited in a liquid transport (SAB-medium) (4). The data regarding age, sex and smoking frequency estimated as cigarette packages per year were collected anonymously from every volunteer participant. Twenty negative controls specimens consisting of swabs impregnated with sterile phosphate buffered saline (PBS) were taken for this study and run in parallel to saliva specimens.

### Saliva Sample Culture

For each sample, a tenfold cascade dilution from 10^−1^ to 10^−6^ was performed in sterile Dulbecco's phosphate buffered saline (DPBS, Gibco Life Technologies; Paisley, United Kingdom) which maintained the pH and osmotic pressure in the cells. The dilutions were carried out in order to isolate the different strains developed subsequently. For each batch of 5 samples, two negative controls containing non-inoculated DPBS were run in parallel. After the dilutions were carried out, each dilution was spread with a rake on Columbia agar containing colistin and nalidixic acid (COS-ANC, bioMérieux, Marcy-l'Etoile, France) incubated at 37°C for 24 h under aerobic conditions. Colonies were sub-cultured and isolated on COS-ANC medium (one COS-ANC culture dish for each transplanted colony) and incubated at 37°C for 24 h in order to obtain pure culture. This protocol was designed to isolate Gram-positive bacteria and avoid contamination by other bacteria forming the oral microbiota (5).

### MALDI-TOF-MS Identification

For each plate, five colonies were tentatively identified by using matrix-assisted laser desorption/ionization mass spectrometry (MALDI-TOF-MS) as previously described (7). Each colony was deposited on a spot of the spectrometer plate by means of a sterile micro-pipette cone and each spot was coated with 1 μL of a matrix solution consisting of saturated α-cyano-4-hydroxycynnamic acid or HCCA (Sigma, Lyon, France), 50% acetonitrile, 25% trifluoroacetic acid, or TFA (Aldrich, Dorset, UK) and 25% HPLC grade water for Hight Purity Liquid Chromatography (VWR, Strasbourg, France). After drying in ambient air, the target plate was introduced into the MALDI-TOF Microflex LT^®^ mass spectrometry device (Bruker Daltonics, Bremen, Germany). Each spot was then analyzed with the help of the FlexControl acquisition software version 3.4 and MALDI Biotyper Compass Analysis Software version 4.1.80 (MBT Compass) (7).

### Statistical Analyses

To test whether tobacco smoking would influence the number of species present in the saliva, we used the generalized linear model binomial function under software R. We used the function R: glm (Formula = PCR 16S~statut + Age + sexe, Family = binomial, data w).

## Results

A total of 90 saliva specimens collected from 90 different individuals comprised of 19 tobacco smokers and 71 non-smokers were investigated specifically for the presence and diversity of Gram-positive bacteria using a routine culture and identification protocol. In all these experiments, the negative controls, which have been manipulated strictly in parallel to tested specimens, remained sterile. A total of 19 Gram-positive bacterial species were cultured in the entire population of 90 individuals. More precisely, 0 to 7 (2.01 ± 1.15) different Gram-positive bacterial species were cultured per saliva specimen. Indeed, saliva specimens remained sterile in nine individuals including six males and three females; and in four tobacco smokers and five non-smokers (Table 1; Figure 1). We observed no difference in the species with respect to the age of the individual (*P*-value, 0.37).

**Table 1:** Diversity of Gram-positive bacteria cultured in the saliva collected from 90 consecutive disease-free individuals comprised of 19 tobacco smokers and 71 non-smokers.

**Sample category**	**Sample number**	**The mean bacterial species by sample category**	**Standard deviation**
Total sample	90	2.01	1.15
Smoker	19	1.47	1.07
Non-smoker	71	2.15	1.13

**Figure 1:** Number of bacterial species found in tobacco smokers and non-smokers. The histogram is showing the mean number of bacterial species accordingly to tobacco smoking/non-smoking status. In blue characters: Total number of samples; in red characters: total number of smoker samples; in green characters: total number of non-smoker samples.

A total of 18 different Gram-positive bacterial species were cultured in males vs. 15 different species in females, with 15 species being isolated in both groups, yet the difference was not significant (*P*-value, 0.17) (Table 2; Figure 2). Accordingly, 2.06 ± 1.23 different Gram-positive bacterial species cultured per sample in males did not significantly differ from 1.77 ± 1.03 species per sample in females (*P*-value, 0.1723) (Table 2; Figure 2).

**Table 2:** Diversity of Gram-positive bacteria cultured in the saliva collected from 90 consecutive disease-free individuals comprised of 62 males and 28 females.

**Sample category**	**Sample number**	**The mean bacterial species by sample category**	**Standard deviation**
Total sample	90	2.01	1.15
Male	62	2.06	1.23
Female	28	1.77	1.03

**Figure 2:** Number of bacterial species found in males and females. The histogram is showing the mean number of bacterial species accordingly to males/females status. In blue characters: Total number of samples; in red characters: total number of sample in male patients; in green characters: total number of samples in female patients.

A total of nine different Gram-positive bacterial species were cultured in 19 tobacco smokers vs. 18 different species in 71 non-smokers (*P*-value, 0.016), with nine species being isolated in both groups (Figure 3). Indeed, all the species cultured from the tobacco smokers' specimens have also been cultured in non-smokers. Accordingly, 1.47 ± 1.07 different Gram-positive bacterial species cultured per sample in tobacco smokers did not significantly differ from the 2.15 ± 1.12 species per sample in non-smokers (*P*-value, 0.16) (Table 2).

**Figure 3:** Number of bacterial species accordingly to status tobacco smokers/non-smokers. X-axis: name of the isolated bacterial species; y-axis: number of isolated bacterial species. The color codes represent the status smokers/non-smokers.

## Discussion

We are reporting on the repertoire of Gram-positive aerobic bacteria in the oral fluid using routine specific isolation and culture and MALDI-TOF-MS to identify bacterial species. The fact that all the negative controls run in parallel with saliva specimens remained negative authenticated the results we reported.

In this study, a total of 19 different Gram-positive bacteria belonging to six genera *Streptococcus, Staphylococcus, Gemella, Granulicatella, Actinomyces*, and *Rothia* were cultured in the oral fluid collected from 90 individuals. Our observations of the overall saliva microbiota concur with previous investigations which used culture-independent methods including metagenomics (8–10); and culture (2, 11, 12). It is noteworthy that our study retrieved by culture some major human pathogens. In particular, *Streptococcus mitis, Streptococcus oralis*, and *Streptococcus sanguinis* are part of the *Streptococcus viridans* group, which is a heterogeneous group of pathogenic streptococci present in the respiratory tract (13). *S. sanguinis* is known to cause endovascular infections (14). *S. pneumoniae* is known to cause otitis, pneumonia and meningitis (15). Thus, most of the bacterial species identified here in the oral fluid are potentially pathogenic species. In particular, culture of *Streptococcus australis* is also remarkable because this species is generally found in children (16). Here *S. australis* was isolated from two adults, a 31-year-old man and a 28-year-old woman. Indeed, one previous isolate *S. australis* strain FRStet12 was also cultured from adult individuals in France, yet from pooled saliva specimens leaving unknown any biographical data regarded the carrier(s) (17). *S. australis* is colonizing the respiratory tract of adult patients diagnosed with cystic fibrosis (18, 19). Also, one case of *S. australis* meningitis was firmly documented in a 77-year-old male patient in France by 16S rRNA gene and *sod*A gene PCR-sequencing in the cerebrospinal fluid; and isolation and culture from two blood cultures (20).

In addition to previous studies, the results here reported showed that tobacco smoking reduced the diversity of saliva Gram-positive bacterial species from 18 in non-smokers down to seven in smokers. As all the species cultured in smokers were also cultured in non-smokers, these results suggest that tobacco smoking has some deleterious effects on the 12 species which have not been cultured in smokers. In particular, the pathogen *S. pneumoniae* was uniquely found in non-smokers in agreement with previous data (21, 22). A recent study using mouth wash specimen and 16S rRNA gene variable V3-V4 region sequencing, found no significant difference as for streptococci, between tobacco-smokers and non-smokers (5). However, this study relied on PCR-based amplification, and was not able to differentiate dead from alive streptococci, as we did.

Some studies on the influence of tobacco smoking on microbial diversity of the oral microbiota using molecular methods have shown a negative influence of smoking on the occurrence of microbial dysbiosis in the oral microbiota (22–24). These results are consistent with our results on the influence of smoking on streptococcal populations in the saliva.

There are several potential mechanisms by which tobacco smoking may alter oral microbial ecology, including increasing the acidity of saliva, depositing many toxicants found in cigarette smoke, depleting oxygen, antibiotic effects, influencing bacterial adherence to mucosal surfaces, and impairing host immunity (22). All these reported elements may favor the survival and development of streptococci, as observed in the present study.

The present study, incorporating only 90 individuals in only one center, warrants confirmation in other centers to overcome any recruitment bias, which may have occurred here. If so, the biological significance of tobacco smoking would have to be explored to assess whether tobacco smoke inhibits the growth of the species specifically found in non-smokers.

## Data Availability

The raw data supporting the conclusions of this manuscript will be made available by the authors, without undue reservation, to any qualified researcher.

## Ethics Statement

All procedures performed in studies involving human participants were in accordance with the ethical standards of the institutional and/or national research committee and with the 1964 Helsinki declaration and its later amendments or comparable ethical standards.

## Informed consent

Informed consent was obtained from all individual participants included in the study.

## Author Contributions

GG performed experiments, interpreted data, and drafted the manuscript. AR performed experiments. ET collected samples and interpreted data. OD performed statistical analyses. MD and GA designed the study, interpreted data, and drafted the manuscript.

### Conflict of Interest Statement

The authors declare that the research was conducted in the absence of any commercial or financial relationships that could be construed as a potential conflict of interest.
